The article "Static and Dynamic Demonstration of the Ecological Level of Ethnic Cultural Industries Based on the Internet of Things and Environmental Responsibility" was retracted in 2023. Reasons: unreliable results or conclusions; concerns about the data; concerns about the peer review; concerns about the citations.

# Static and Dynamic Demonstration of the Ecological Level of Ethnic Cultural Industries Based on the Internet of Things and Environmental Responsibility

**DOI:** 10.1155/2022/5953522

**Published:** 2022-09-29

**Authors:** Weiguang Xie, Shanbo Yu

**Affiliations:** ^1^College of Humanities and Tourism, Yiwu Industrial & Commercial College, Yiwu, 322000 Zhejiang, China; ^2^College of Economics and Management, Jiamusi University, Jiamusi, 154007 Heilongjiang, China

## Abstract

The cultural industry of ethnic minorities carries the wisdom of many ancients. In today's modernization, ethnic minority cultural industry products can still impress people's hearts with exquisite handicrafts, natural materials, and strong culture. The rise in demand for ethnic cultural products will bring about an increase in the demand for raw materials for handmade products, which is bound to have an impact on the environment. This paper is aimed at modeling and analyzing the ecological level of minority cultural industries based on the background of the Internet of Things (IoT) and environmental responsibility. In the experiment, this paper analyzed the ecological level of the traditional fish skin industry by taking the Hezhe people in Heilongjiang as an example. Aiming at the cultural industry of the Hezhe people, this paper selected the fish skin industry as the object of empirical analysis from the fish culture it represents. According to the ecological level of the industry, this paper selected the three first-level indicators of production energy saving level, ecological environmental protection level, and production emission reduction level and its 12 subordinate second-level indicators to model and analyze the fish skin industry of the Hezhe people. The analysis results showed that the industrial ecological level of the Hezhe fish skin industry in the past 16 years reached the standard rate of more than 75%. However, the ecological level index for the three years of 2018, 2019, and 2020 was between 0.3 and 0.5, which indicated that the ecological level in these three years was very low. This was caused by the mechanization of the handicraft industry in recent years.

## 1. Introduction

A nation's culture includes all emotions and attitudes involved in production and life, including material culture and spiritual culture formed in the interaction with the natural environment. The interaction and combination of the two constitute a complex national culture. Material culture is represented by clothing, handicrafts, dwellings, and food; spiritual culture is represented by language, customs, religion, taboo, social class, belief, etc. For cultural products, buyers mainly want to appreciate the special ethnic customs and satisfy their psychology of seeking difference, novelty, knowledge, pleasure, and exploration. Therefore, when cultural products are developed, culture should be regarded as the soul, and innovation should be carried out around it.

The article "Static and Dynamic Demonstration of the Ecological Level of Ethnic Cultural Industries Based on the Internet of Things and Environmental Responsibility" was retracted in 2023. Reasons: unreliable results or conclusions; concerns about the data; concerns about the peer review; concerns about the citations.

Cultural industry is a special form of cultural development, which links culture and economy together. Cultural exchange, dissemination, and development are realized, and economic benefits are obtained. The Hezhe people have a unique fish culture, which is a production and living culture based on a special natural and geographical environment. This reflects the cultural atmosphere of the combination of humanities and nature. Different from the cultural customs among different ethnic groups is the main advantage of the Hezhe people in developing the cultural industry. The quaint and simple Hezhe customs are packaged into cultural products combined with modern culture, which does not lose its essence and does not highlight the trend. The excavation of cultural connotation must be paid attention to develop the cultural industry. If the industry is simply developed and the infiltration of cultural connotation is not valued, the development of the industry will be too single. The lack of the enrichment of cultural content makes the industrial development lack core competitiveness and stamina. The Hezhe fish culture is the core of developing the cultural industry. Therefore, the Hezhe people should pay attention to taking culture as the center of development while developing the cultural industry. The essence of development culture is the embodiment of competitiveness in the process of industrialization.

Ethnic minorities have a more traditional way of life and older technical skills. Their handmade products have more cultural heritage. For the cultural industry of ethnic minorities, many scholars have conducted researches. Based on sociological theory, Tarlow analyzed the inclusiveness of minority cultural industries and provided suggestions for the development of tourism from traditional industries [1]. Ding et al. used the corpus method to collect cultural industry news in Shanghai, Guangdong, Sichuan, and Shaanxi pilot free trade zones. The corpus was constructed and Python was used to analyze data from the cultural industry [2]. Rahimi et al. aimed at defining sustainability standards for traditional beekeeping in Iran, which was carried out using the three-stage classic Delphi technique [3]. Chen conducted a research on the development of cultural industry in recent years. A new direction for the development of ethnic minority traditional cultural industries was proposed [4]. Based on the collaborative innovation of the government, enterprises, universities, scientific research institutions and users, Wang et al. used the method of case study to analyze the situation of Shanghai's marine cultural industry. He also analyzed the possible deficiencies in talent training and proposed specific measures for talent training in the marine cultural industry [5]. However, their researches were more about the development and promotion of traditional industries. The purpose was to improve the economy of traditional industries. Responsibility for the ecological environment was not considered.

The article "Static and Dynamic Demonstration of the Ecological Level of Ethnic Cultural Industries Based on the Internet of Things and Environmental Responsibility" was retracted in 2023. Reasons: unreliable results or conclusions; concerns about the data; concerns about the peer review; concerns about the citations.

An environment-friendly society has always been the goal pursued by human beings. However, the economy and the environment have always been mutually destructive, which is an antagonistic relationship. There are many scholars who have done researches on the ecologicalization of industry. Based on the green economy theory, Jammoukh et al. used the gray system theory to make a dynamic forecast and analysis of the green development level of the development zone during the “Twelfth Five-Year Plan” period [6]. Yuan et al. used the gray dynamic correlation model to couple the three indicators with the economic growth rate and industrial structure optimization indicators [7]. Guan et al. established a comprehensive soil risk assessment method in industrial and mining areas. Taking a typical industrial and mining area as an example, the soil pollution risk was evaluated quantitatively and spatially [8]. Zhang et al. measured the pollution level of heavy industry and provided suggestions for its ecological construction based on the location of heavy industry [9]. Malshe and Krush focused its attention on the enterprise level. They regarded the production and sales link of the enterprise as a whole and designed the ecological evaluation indicators for the overall process of production and sales of products [10]. However, their researches were too broad. Specific cases have not been analyzed and the underlying operating principles have not been described.

The main innovations of this paper are combining the Internet of Things and the awareness of environmental ecological responsibility; the traditional cultural industries of ethnic minorities are analyzed from the perspective of environmental protection. In terms of analysis, the Hezhe fish skin industry is taken as the object of empirical analysis, which is specific to the meticulous industry. This kind of analysis is more targeted and has certain reference for the subsequent ecological development of the cultural industry. And in the analysis, the data obtained from the actual visit is used for analysis, which is very important for the verifiability and reliability of the results.

The article "Static and Dynamic Demonstration of the Ecological Level of Ethnic Cultural Industries Based on the Internet of Things and Environmental Responsibility" was retracted in 2023. Reasons: unreliable results or conclusions; concerns about the data; concerns about the peer review; concerns about the citations.

## 2. Minority Cultural Industries

### 2.1. Internet of Things and the Cultural Industry of Ethnic Minorities

Undoubtedly, the Internet of Things can bring huge economic and social benefits to the cultural industry of ethnic minorities, which is a key strategy for grasping the initiative of science and technology in the 21st century [11]. As shown in Figure 1, the application of the Internet of Things has been involved in all aspects of life.

Now, the Internet of Things is based on the Internet and extends the “tentacles” of the network to “everything.” Therefore, problems such as information security, information explosion, and digital divide brought by the Internet may become more serious on the Internet of Things. The disruptive and harmful nature of the Internet of Things will be even more profound. This is completely contrary to the original intention of the Internet of Things design. Therefore, at the beginning of the full application of the Internet of Things, it is necessary to study its possible social impacts, especially negative impacts. The economic and social benefits brought by the Internet of Things need to be timely fed back, improved, and expanded [12]. The Internet of Things can connect with any item in time and space, which makes the Internet of Things reach a new dimension, as shown in Figure 2.

As a material form of information culture, it is based on the “value” brought by information technology. This is the materialized basis of the entire information culture, which provides a solid humanistic environment for the circulation of information. Information economy and information technology are the main contents of information culture as material form [13, 14]. At the level of the information economy and information technology, the Internet of Things may have the following effects on culture:

Unemployment problem will be serious: the Internet of Things uses informatization as the means to promote the development of the information economy, which is mainly reflected in cost savings. It can not only achieve precise and meticulous control of all aspects of the economy but also reduce useless work. However, unemployment problems will follow. If the smart grid is implemented, meter readers will have nothing to do. Smart farming will drive more farmers off the land, and smart healthcare will drive more doctors off. Although the development of the Internet of Things can spawn many new industries and provide more jobs, it is very difficult to retrain those who have worked in familiar jobs for many years.

The development path of green economy is tortuous: the Internet of Things itself is a typical representative of green economy and low-carbon economy, which is also an important step in the transformation of information culture to “green culture.” The Internet of Things is aimed at the green economy. By providing a series of applications such as smart buildings, smart cities, and smart environmental protection, the goals of energy conservation, emission reduction, and resource waste reduction can be achieved. In the construction of smart buildings and smart cities, how will the original infrastructure be handled? Due to the diversity of the original infrastructure, it is not only time-consuming and labor-intensive to transform on the original basis, but also it is impossible to know whether the expected effect can be achieved. If “breaking the old and building the new” is implemented, it will cause even greater waste. How to start a green economy? How can this be considered a green economy?

The article "Static and Dynamic Demonstration of the Ecological Level of Ethnic Cultural Industries Based on the Internet of Things and Environmental Responsibility" was retracted in 2023. Reasons: unreliable results or conclusions; concerns about the data; concerns about the peer review; concerns about the citations.

### 2.2. Hezhe Fish Culture

The fish culture of the Hezhe nationality refers to the cultural summation composed of the material culture created by the Hezhe nationality in production and life mainly based on the skin of fish, eating fish meat, and making fish skin handicrafts and spiritual culture with fish as totem belief under the natural conditions of the cold climate and abundant water in the early northeast. Fish culture is the tangible fish pictures, fish objects, and intangible fish customs and fish beliefs, which carry the wisdom and spirit of the Hezhe people and represent the life attitude of the simple Hezhe people who love, fear, and worship nature. This has important reference significance for coordinating the contradiction between man and land in today's society [15]. As shown in Figure 3.

Among the many Hezhe fish cultures, fish skin products are the most suitable for trading in the market as cultural products. Among them, there are many classifications of fish skin products, such as fish skin clothes, trousers, fish skin straw sandals, fish skin ornaments, and fish skin paintings. Among them, the fish skin coat is the most representative. Making fish skin into clothes is a very complicated job, which requires a series of delicate processes such as skin selection, peeling, drying, hammer pressing, stitching, cutting and stitching, and rust decoration. Skin selection is to classify different types of fish skins. The soft skin of the fish is used to make clothes, and the thin and tough skin is used to make the fish skin line. Peeling is to peel off a whole piece of fish skin with scales, which is very difficult. The skin of the fish should be dried and dehydrated without losing its toughness. After peeling the fish skin, dry the skin by the fire, roll the skin tightly, put it in a wooden groove about 5 cm long and 2.5 cm wide, beat it with a sharp-free iron axe, or a special wooden axe, or put press repeatedly under the wooden rolling knife to soften the leather. You can also put cornmeal in the skin, which can remove the oil on the fish skin. Whether the fish skin clothes are soft, tough, and strong is closely related to the process of handling the skin [16]. After cutting, sewing, and decoration, the production of a fish skin garment is initially completed. The production process of fish skin clothes is complicated. At this stage, the production of fish skin products is all done by hand and machine production has not yet been popularized. Some fish skin industry products are shown in Figure 4.

The article "Static and Dynamic Demonstration of the Ecological Level of Ethnic Cultural Industries Based on the Internet of Things and Environmental Responsibility" was retracted in 2023. Reasons: unreliable results or conclusions; concerns about the data; concerns about the peer review; concerns about the citations.

### 2.3. Evaluation Model of Ecological Level

There are many methods for evaluating industrial ecologicalization. In the commonly used industrial ecologicalization evaluation models, whether the subjective weighting method or the objective weighting method is used to determine the index weight has certain limitations. On the basis that the advantages and disadvantages of various evaluation models are compared, and the application scope of each model is analyzed, this paper refers to the existing research results of other scholars and combines the improved information entropy with the principal component analysis method to evaluate the industrial ecological level. The model not only integrates subjective and objective factors, but also conducts specific analysis on each criterion layer in the index system. This enables the development status of the coking industry to be analyzed in more detail [17].

Information entropy is a basic concept of subordinate information theory, which is used to measure the amount of information. It is assumed that a system *X* may appear in several different states *x*_1_, ⋯, *x*_*n*_, *p*(*x*_*i*_) represents the probability of the occurrence of *x*_*i*_(*i* = 1, 2, ⋯, *n*) states, then the information entropy *H*(*X*) of the system is defined as

(1) $$\begin{array}{c} H\left(X\right)=-\overset{n}{\underset{i=1}{\sum }}p\left(x_{i}\right)\log\left(p\left(x_{i}\right)\right). \end{array}$$

In the formula, 0 ≤ *p*(*x*_*i*_) ≤ 1 and ∑_*i*=1_^*n*^*p*(*x*_*i*_) = 1. When *p*(*x*_*i*_) = 0, *p*(*x*_*i*_)log(*p*(*x*_*i*_)) = 0.

Information entropy is a method used to measure the ordering level of a system; the information entropy value of a system is inversely proportional to the degree of order of the system. The larger the information entropy value, the more disordered the system is. The information entropy obtains the index weight value through the operation of the data value of each index, which does not consider the influence of subjective factors on the evaluation object at all. The weight of each index is a reflection of the amount of effective information it contains. Therefore, the weights calculated by the information entropy method cannot fully reflect the importance of the indicators. The empirical factor also has a decisive effect on the indicator weight [18]. In this paper, experts' understanding of the importance of each index is added to the information entropy calculation. By constructing an expert decision reciprocal matrix, the row sum normalization method and the principle of minimum information entropy are used to improve and supplement the weight determined by traditional information entropy. Finally, the optimal solution of the comprehensive weight is obtained.

The article "Static and Dynamic Demonstration of the Ecological Level of Ethnic Cultural Industries Based on the Internet of Things and Environmental Responsibility" was retracted in 2023. Reasons: unreliable results or conclusions; concerns about the data; concerns about the peer review; concerns about the citations.

In this paper, the three first-level indicators are, respectively, established by the information entropy method to establish the evaluation model. 3 first-level index rankings are obtained. Assuming that a first-level indicator contains *m* H-level small indicators, then a second-level indicator is determined by a third-level indicator matrix. The specific calculation steps of each second-level indicator are as follows:

1 secondary indicator *k* (*k* = 1, 2, ⋯, *p*) contains *n* enterprise samples and *m* attribute indicators, which constitute the H-level indicator matrix *A*_*k*_:

(2) $$\begin{array}{c} A_{k}=\left(\begin{array}{ccc} a_{11} & \cdots & a_{1m}\\ \vdots & \ddots & \vdots \\ a_{n1} & \cdots & a_{nm} \end{array}\right). \end{array}$$

In the formula, *p* is the number of secondary indicators, *n* is the participating enterprises, *m* is the number of H-level indicators included in the *k*-th secondary indicator.

Positive and negative indicators are defined. The positive index *a*_*ij*_^+^ ≥ 0 indicates that the larger the specific data value of the index, the better the level of industrial ecologicalization; the inverse index *a*_*ij*_^−^ ≥ 0 indicates that the smaller the specific data value of the index, the better the level of industrial ecologicalization. In order to ensure the consistency of each index in the evaluation of industrial ecologicalization and in the calculation of information entropy, it is necessary to standardize the positive and inverse indicators [19].

Positive attribute index normalization:

(3) $$\begin{array}{c} r_{ij}=\frac{a_{ij}^{+}-\min\left(a_{ij}^{+}\right)}{\max\left(a_{ij}^{+}\right)-\min\left(a_{ij}^{+}\right)}. \end{array}$$

Inverse attribute index normalization:

(4) $$\begin{array}{c} r_{ij}=\frac{\max\left(a_{ij}^{-}\right)-a_{ij}^{-}}{\max\left(a_{ij}^{-}\right)-\min\left(a_{ij}^{-}\right)}. \end{array}$$

After standardization, the decision matrix *R*_*k*_ of the *k*-th secondary indicator is obtained.

(5) $$\begin{array}{c} R_{k}=\left(\begin{array}{ccc} r_{11} & \cdots & r_{1m}\\ \vdots & \ddots & \vdots \\ r_{n1} & \cdots & r_{nm} \end{array}\right). \end{array}$$

The entropy *E*_*j*_ of the attribute index *j* is:

(6) $$\begin{array}{c} E_{j}=-k\overset{n}{\underset{i=1}{\sum }}r_{ij}\ln\left(r_{ij}\right). \end{array}$$

Information bias:

(7) $$\begin{array}{c} d_{j}=1-E_{j}. \end{array}$$

The weight of an index *j* refers to the degree of influence of the index *j* on the evaluation object. The so-called weight represents the decisive quantitative performance of the evaluation index in the overall evaluation. The size of the weight value of the indicator is proportional to the influence of the indicator on the evaluation result. The weight of the indicator *j* is

(8) $$\begin{array}{c} \omega_{j}^{1}=\frac{d_{j}}{\sum_{j=1}^{m}d_{j}},\\ =\frac{1-E_{j}}{m-\sum_{j=1}^{m}E_{j}}. \end{array}$$

From Formula (2) to Formula (8), the weight value obtained by the information entropy is obtained. However, it cannot fully represent the importance of indicators. The experience factor of experts in the relevant field is also very important to the decision result. Therefore, the information entropy needs to be improved. In the following part, by constructing the expert decision reciprocal matrix, the row sum normalization method and the most information entropy principle are adopted, the expert's experience factor is incorporated into the information entropy, and the optimal solution of the weight is obtained [20].

The article "Static and Dynamic Demonstration of the Ecological Level of Ethnic Cultural Industries Based on the Internet of Things and Environmental Responsibility" was retracted in 2023. Reasons: unreliable results or conclusions; concerns about the data; concerns about the peer review; concerns about the citations.

According to the reciprocal matrix given by the expert, the row sum normalization method is used to calculate the weight vector of the evaluation index

(9) $$\begin{array}{c} \omega_{j}^{2}=\frac{\sum_{j=1}^{n}a_{ij}}{\sum_{k=1}^{n}\sum_{j=1}^{n}a_{kj}}. \end{array}$$

The combined weight, *ω*_*j*_ is obtained by the weight *ω*_*j*_^1^ calculated by the information entropy, and the weight *ω*_*j*_^2^ is calculated by the expert opinion. According to the principle of minimum information entropy, the formula is

(10) $$\begin{array}{c} \min E=\overset{m}{\underset{i=1}{\sum }}\omega_{j}\ln\frac{{\left(\omega_{j}\right)}^{2}}{\omega_{j}^{1}\omega_{j}^{2}}. \end{array}$$

When min*E* satisfies the minimum, the optimal solution can be obtained. The Lagrange multiplier method is used to construct the function to optimize the solution, and the formula can be obtained:

(11) $$\begin{array}{c} \omega_{j}=\frac{\sqrt{\omega_{j}^{1}\omega_{j}^{2}}}{\sum_{i=1}^{m}{\left(\omega_{j}^{1}\omega_{j}^{2}\right)}^{0.5}}. \end{array}$$

It can be seen from the calculation that only when the part *ω*_*j*_ is equal to the geometric mean of *ω*_*j*_^1^ and *ω*_*j*_^2^, the min*E* can be minimized, and the optimal solution can be obtained, and thus, the comprehensive weight of each evaluation index can be obtained.

The article "Static and Dynamic Demonstration of the Ecological Level of Ethnic Cultural Industries Based on the Internet of Things and Environmental Responsibility" was retracted in 2023. Reasons: unreliable results or conclusions; concerns about the data; concerns about the peer review; concerns about the citations.

The evaluation value of the secondary index is

(12) $$\begin{array}{c} Z_{i,k}=\overset{m}{\underset{j=1}{\sum }}\omega_{j}r_{ij}. \end{array}$$

By repeating the steps, the secondary indicator matrix of the 3 secondary indicators is obtained:

(13) $$\begin{array}{c} Z_{n,p}=\left(\begin{array}{ccc} z_{11} & \cdots & z_{1p}\\ \vdots & \ddots & \vdots \\ z_{n1} & \cdots & z_{np} \end{array}\right). \end{array}$$

The principal components of the primary indicators are used to analyze the evaluation model.

The secondary index matrix *Z*_*n*,*p*_ is subjected to principal component analysis, and the correlation coefficient matrix *R* is calculated.

The *p* eigenvalues of *R* are computed:

(14) $$\begin{array}{c} \lambda_{1}\geq \lambda_{2}\geq \cdots \geq \lambda_{p}\geq 0. \end{array}$$

The corresponding eigenvector is

(15) $$\begin{array}{c} e_{j}=\left(l_{1j},l_{2j},\cdots ,l_{pj}\right). \end{array}$$

The variance contribution rate is calculated:

(16) $$\begin{array}{c} \alpha_{i}=\frac{\lambda_{i}}{\sum_{k=1}^{p}\lambda_{k}}. \end{array}$$

The variance contribution rate is sorted in descending order, if the cumulative variance contribution rate of the first m indicators satisfies the following:

(17) $$\begin{array}{c} \alpha_{svm}=\overset{m}{\underset{k=1}{\sum }}\alpha_{k}\geq 85\%. \end{array}$$

Then, it is considered that the *m* principal components can comprehensively reflect *p* indicators.

The principal components of a sample of *n* years are computed:

(18) $$\begin{array}{c} M_{i,j}=Z_{n,p}\times {\left[e_{1},e_{2},\cdots ,e_{p}\right]}^{l}. \end{array}$$

The first *m* principal components are selected, and the first-level indicators are obtained by calculation

(19) $$\begin{array}{c} F_{i}=\overset{m}{\underset{i,j}{\sum }}\alpha_{j}M_{i,j}. \end{array}$$

*F*_*i*_ is sorted, that is, the comprehensive evaluation ranking is obtained.

## 3. Demonstration of the Level of Industrial Ecologicalization

### 3.1. Natural Ecology of the Hezhe People in Raohe County

The biotechnological methods of the Hezhe people seem to be used as national symbols. Living along the river and surrounded by mountains and forests endow the Hezhe people with good conditions for fishing and hunting. Raohe County governs the area along the west bank of the Ussuri River, surrounded by mountains and rivers. The mountains in the south and west belong to the Wanda Mountains, which are mostly forested with birch, linden, oak, pine, poplar, elm, willow, and other trees. [21] Forests account for more than 79% of the county's land area, and there are many wild animals such as tigers, bears, deer, wild boars, and wolves, as well as fine-haired beasts such as nettles, foxes, weasels, and Shaw. In the north, the vast fields of the Naoli River, the Bilayin River, the Nongjiang River, and the Qili River form an area where the rivers and canals are crisscrossed in the lower reaches of the three rivers. These water towns are rich in fish such as maha, carp, crucian carp, ham, catfish, mandarin fish, and fine lin. These natural conditions are suitable for the Hezhe people hunting and fishing production. From the perspective of latitude and longitude, Raohe County is located in the frigid zone. The lowest temperature over the years is below minus 35 degrees Celsius and the highest temperature is above 30 degrees Celsius. The icing period starts from late October to mid-November on the solar calendar every year, and the ice-releasing period starts from mid-May. The farming period is about six months from late April to early October. The climate here is moderately sunny and rainy, which is suitable for agricultural production. The soil here is fertile, generally clay or clay-sand mixed with humus, which is suitable for cultivating paddy fields [22, 23].

The article "Static and Dynamic Demonstration of the Ecological Level of Ethnic Cultural Industries Based on the Internet of Things and Environmental Responsibility" was retracted in 2023. Reasons: unreliable results or conclusions; concerns about the data; concerns about the peer review; concerns about the citations.

Feeding on fish and animal meat and using fish and animal skins as raw materials for clothing is a true portrayal of the life of the Hezhe people. From the beginning of spring fishing, the women began to process fish skins. Until the fall, the skins needed for the year are picked out to make clothes and leather goods. Animal skins are also processed in spring, summer, and autumn. And these processed products are used to make clothing for winter hunting.

Various fish skins have different uses. For example, fathead fish and pike skin can be used as fish skin lines and pants. Fish skins such as white head fish, jellyfish, salmon, and tangled fish can be used as lepers; tartar can also be used as hand stuffy son. Carp skin and fish skin can be used as clothes and trousers. The wrapping fish skin will not become moldy after being soaked in water, so the clothes made of wrapping fish skin are worn when fishing in summer, and other clothes made of fish skin are worn in winter. Animal hides also have varying degrees of use due to their different properties. Dog skins are mainly used to make quilts, mattresses, coats, hats, etc. Deerskin can be used to make all kinds of clothes and cigarette pockets. Bear skins and boar skins can be used as boots and mattresses. [24]

The article "Static and Dynamic Demonstration of the Ecological Level of Ethnic Cultural Industries Based on the Internet of Things and Environmental Responsibility" was retracted in 2023. Reasons: unreliable results or conclusions; concerns about the data; concerns about the peer review; concerns about the citations.

### 3.2. Selection of the Evaluation Index System for the Ecological Level of the Hezhe Fish Skin Industry

To achieve ecological development, the Hezhe fish skin industry includes not only economic factors, but also environmental, ecological, humanistic, and other factors. Therefore, this paper cannot only focus on one aspect in the process of researching the problem, but must consider it comprehensively. Therefore, in the design of the indicator system, three major categories and twelve subcategories are divided [25].

When the data is standardized, data is mainly obtained from the National Bureau of Statistics and a small amount of data is obtained from enterprise surveys. Then different categories of data are combined for standard processing to obtain various indicator data; at the same time, according to the influence degree of each data on ecologicalization, different index weight coefficients are set, an ecological evaluation model is established and relevant ecological data indicators are calculated.

In the normalization of the index data, the methods of forwardization and dimensionlessization are used. The indicators that positively promote the ecological level of the Hezhe fish skin industry are positive indicators, and this indicator includes data related to waste treatment. And the higher the data, the higher the standard of ecological level. Inverse indicators have a negative effect on the Hezhe fish skin industry. For example, the higher the exhaust emission, the lower the ecological level. This is a inverse indicator. When determining the index system, there must be a distinction between forward and reverse, otherwise, the data cannot be calculated scientifically. The forward processing is to take the reciprocal of the reverse index, and this forward processing is conducive to the dimensionless analysis of the index. Some indicators have different data and defined dimensions, so comparisons cannot be made. Therefore, the affected amount must be eliminated [26, 27].

As shown in Table 1, the expert scores are 1, 2, 4, 6, and 8 according to the scale of 1-9, indicating the importance of the *ω*_*i*_ index relative to *ω*_*j*_Table 1 lists the specific scale table.

After that, the calculation and judgment parameters are shown in Table 2.

Finally, the data is input into SPSS software, and the weight of each secondary indicator is obtained as shown in Table 3.

Then combined with the actual situation, the three first-level indicators are analyzed separately.

### 3.3. Production Energy Saving Level Index and Secondary Index

As shown in Figure 5, the correlation of the production energy saving level indicators can be seen. During the current study period, the energy consumption per unit of Gross Domestic Product (GDP) showed a steady upward trend. There are two indicators: energy consumption per unit of GDP. Both the comprehensive index and the electricity consumption index per unit of GDP belong to the growth stage, which tends to rise steadily. It can be seen from the previous investigation that the electricity consumption of million industrial output value can only be said to be much higher than that of the other three, with an exponential growth. That said, during this period, the fish skin industry has made significant progress in improving the efficiency of electrical energy utilization. However, the index of water consumption per unit of GDP is one of the indicators studied. During this period, the fish skin industry had a high demand and dependence on water resources. At the same time, there is no optimal use of water resources. The significant increase in the index in 2018 shows that the energy conservation and emission reduction work adopted in recent years has achieved remarkable results. The dependence on water resources is reduced, and the utilization rate of water resources is improved. The energy consumption elasticity index has also increased significantly from the beginning of the study to the present, from -0.065 in 2011 to 0.139 in 2020. The energy-saving level index of fish skin industry production is shown in Figure 5.

The article "Static and Dynamic Demonstration of the Ecological Level of Ethnic Cultural Industries Based on the Internet of Things and Environmental Responsibility" was retracted in 2023. Reasons: unreliable results or conclusions; concerns about the data; concerns about the peer review; concerns about the citations.

From Figure 5, it can be concluded that the energy-saving level of Hezhe fish skin industry production from 2011 to 2020 is rising, but there are different levels of growth every year. Especially in recent years after 2016, there has been a more rapid growth. The reason for this situation is related to the transformation of the economic growth pattern after 2016. The initial extensive economic growth has now become dependent on scientific and technological progress and human resources. The policies of the relevant functional departments of Heilongjiang Province have strongly supported the industry, and the state has also subsidized it. The energy efficiency of enterprises has been improved, and the level of the fish skin industry has been promoted.

### 3.4. Ecological and Environmental Protection Level Index and Secondary Index

From the data in Figure 6, it can be concluded that from 2011 to 2020, the proportion of environmental protection output value continued to show an upward trend year by year. But there have also been two particularly volatile years in the process, that is, 2012 and 2019. Although there have been some fluctuations in the past two years, it does not affect the overall development trend of growth. What really matters is the right question reflected behind it. Society is constantly developing and progressing. It can be found that the smallest index among the three indices in 2011 is -0.254. It is also because in the early stage of research and development, the focus of entrepreneurs and investors is not one aspect. From 2011 to 2020, various indicators are constantly changing. Among them, the rapid growth in 2018-2019 also reflects the good foundation of ecological environmental protection, so that this rapid and steady upward trend can be obtained. By 2018, the metric is higher than the other two indices. In the course of development in the past ten years, Heilongjiang Province has been increasing its investment in this field. From 2011 to 2020, the trend of the waste disposal rate index can also be used to judge its efforts in this regard, rising from -0.231 in 2011 to 0.135 in 2020. The ecological and environmental protection level indicators of Hezhe fish skin industry over the years are shown in Figure 6.

The article "Static and Dynamic Demonstration of the Ecological Level of Ethnic Cultural Industries Based on the Internet of Things and Environmental Responsibility" was retracted in 2023. Reasons: unreliable results or conclusions; concerns about the data; concerns about the peer review; concerns about the citations.

By analyzing the information in Figure 6, it can be concluded that during the period from 2011 to 2020, the entire environmental protection index continued to show a steady, rising, and increasing trend, which rise from -0.635 in 2011 to 0.512 in 2020. Among them, the period from 2017 to 2018 has developed rapidly, which reflects the actual situation that the government is vigorously promoting the concept of environmental protection. However, from 2018 to 2019, the development is relatively slow and not as obvious as before. It is because after the development reaches a certain level, the period of rapid growth has passed. Environmental protection work will be a long-term process. The faster development in 2020 is also related to less pollution emissions during the epidemic prevention and control period.

### 3.5. Production Emission Reduction Level Index and Secondary Index

From the data in Figure 7, the corresponding index changes and trends can be seen. The rapid rise in the wastewater discharge rate index from 2011 to 2020 shows that the work done by the industry has not been effective in reducing wastewater discharge. In 2020, the proportion of wastewater discharge per unit of output value will increase by 0.2158, which shows that more work and efforts need to be done in wastewater discharge. The overall exhaust emission rate is on the rise. The small decline around 2012 did not affect the overall upward trend. The growth rate of this indicator has accelerated around 2019, and attention should be paid to increasing the control of exhaust emissions. From 2011 to 2020, waste emissions showed a steady upward trend. Affected by economic development in 2012, it fell slightly and then continued to rebound. Although the overall development of wastewater compliance rate is relatively unstable, it developed rapidly from 2014 to 2017, and reached a maximum of 0.098 in 2018. This rapid growth declined significantly in 2019. This is in an unstable state. Although it rose to 0.115 in 2020, this unstable state did not reach the highest value in 2018 but remained basically within the stable state. The exhaust gas emission compliance rate rose from -0.133 to 0.086, showing an upward trend. This shows that the government has done a lot of work on exhaust emissions. The annual emission reduction level indicators of Hezhe fish skin industry are shown in Figure 7.

The article "Static and Dynamic Demonstration of the Ecological Level of Ethnic Cultural Industries Based on the Internet of Things and Environmental Responsibility" was retracted in 2023. Reasons: unreliable results or conclusions; concerns about the data; concerns about the peer review; concerns about the citations.

By analyzing the information in Figure 7, it can be concluded that during the period from 2011 to 2020, the overall level index is an increasing trend with an overall upward trend. Through this trend, it can be shown that a number of industries have begun to carry out continuous research and rationalization of transformation and upgrading in this regard. It rose from -0.791 in 2011 to 0.697 in 2020. Then from 2011 to 2020, the emission reduction index showed a trend of stable development and a gradual increase, that is to say, the government is constantly increasing its capital investment in this area. During the period from 2014 to 2018, there has been rapid development. After 2018, although there is a trend of growth, it is less obvious than other years.

## 4. Demonstration of Hezhe Fish Skin Industry

The data are mainly derived from the actual survey of fish skin industry enterprises. Through the statistics and sorting of the relevant indicators of the daily fish skin industry for 16 years, the data information within 16 consecutive days is selected. The daily data is composed of 16-dimensional features, and the data of each dimension's features after dimensionless processing is shown in Figure 8. There are large differences in units and data sizes between indicators. In order to achieve unified processing, the data can be dimensionless processed first. The entropy weight method is used to determine the principle of their respective weights, so that the final index data dimensionless result is between 0.1-0.95.

Humans will select specific parts to focus on when processing images, which is the so-called attention mechanism. This mechanism is also used in computer and machine vision. In the face of complex scenes, a global overview is firstly browsed, and then a centralized observation is performed according to the algorithm. This mechanism can also be well applied to the determination of indicator weights. In this paper, the method of attention mechanism is applied to the data recording of the ecologicalization of the Hezhe fish skin industry. The weight value assigned to each index feature is determined according to the size of the attention weight and multiple features can be better integrated. The ecological level of evaluation based on the feature can be achieved, as shown in Figure 9.

The article "Static and Dynamic Demonstration of the Ecological Level of Ethnic Cultural Industries Based on the Internet of Things and Environmental Responsibility" was retracted in 2023. Reasons: unreliable results or conclusions; concerns about the data; concerns about the peer review; concerns about the citations.

In the research process of this paper, the evaluation of the fish skin ecosystem should have clear standards and grades. Referring to the relevant literature on ecosystem assessment in the previous theoretical part, this paper divides the grades of fish skin ecosystem security assessment. The corresponding scores are shown in Table 4.

According to the previous analysis and calculation, the ecologicalization of the fish skin industry in Heilongjiang Province is early-warned. By tracking the data, the security level is analyzed. According to the ecological level, when the comprehensive evaluation level of the year reaches level D (less safe) and level C (critical safety), an early warning should be activated to prevent further deterioration of the ecological level. The data from 2005 to 2020 are simulated, and the results are shown in Figure 10.

As shown in Figure 10, the security of the fish skin ecosystem in the past 16 years is not so optimistic. The environmental protection meaning of a large number of traditional workshops is low, and the damage to the environment is getting worse. For large enterprises, the relevant systems are not perfect and environmental issues are not paid enough attention. It can be seen that after 2015, the evaluation level of the system is getting lower and lower, which shows that the ecological problem of the Hezhe fish skin industry is facing great difficulties.

## 5. Conclusions

At present, the Hezhe fish skin industry does not have a complete system, and the development of the cultural industry requires mass production of cultural products in accordance with industrial production standards. The hand-making of Hezhe fish skin products will affect the overall development of the cultural industry. Since fish skin clothing is a finely processed product, it must be made by hand, and it is not recommended to be done by machine. But other fish skin products such as fish skin paintings and fish skin ornaments are easier to complete by machines. Whether it is the economic development of the Hezhe nationality or the protection of traditional culture, cultivating and absorbing a large number of talents is the fundamental guarantee for success. In terms of economy, governments at all levels should provide preferential conditions for some Hezhe people to return to their hometowns to start businesses. For example, the government can contact various large enterprises to provide internship opportunities for Hezhe students, allowing them to learn the advanced management experience of these enterprises. Preferential policies on capital and technology are provided to enable students to return to hometowns to start businesses. These students born and grew up here, and their understanding of the local area and the grasp of local wisdom are naturally better than those brought in from outside. The cultivated phoenix should be allowed to fly back to hometown. In the current transitional period, it is not only necessary to recruit “the businessmen of other countries” and “the capital of other countries,” but also to give greater financial and policy support to those capable people who can establish themselves in the village and lead the villagers to start their own businesses. In addition, in terms of culture, the government should actively cultivate the inheritors of the Hezhe culture and the management talents for the management of the Hezhe culture. Research talents on Hezhe culture should also be absorbed. To develop the fish culture industry, the Hezhe people must take culture as their soul. The distinctive culture of Hezhe needs to be extracted and packaged.

The article "Static and Dynamic Demonstration of the Ecological Level of Ethnic Cultural Industries Based on the Internet of Things and Environmental Responsibility" was retracted in 2023. Reasons: unreliable results or conclusions; concerns about the data; concerns about the peer review; concerns about the citations.

## Figures and Tables

**Figure 1:** Application of the Internet of Things.

**Figure 2:** The new dimension of the Internet of Things.

**Figure 3:** Hezhe fish culture.

**Figure 4:** Fish skin industry products.

**Figure 5:** Index of production energy saving level.

**Figure 6:** Ecological environmental protection level index.

**Figure 7:** Emission reduction level index.

**Figure 8:** Dimensionless data of fish skin ecosystem for 16 consecutive days.

**Figure 9:** Attention mechanism.

**Figure 10:** System ecological security evaluation results in the past 16 years.

**Table 1:** Reciprocity scale column.

Serial number	Compare	*b*_*ij*_
1	*ω*_*i*_ is as important as *ω*_*j*_	1
2	*ω*_*i*_ is slightly more important than *ω*_*j*_	2
3	*ω*_*i*_ is obviously more important than *ω*_*j*_	4
4	*ω*_*i*_ is more important than *ω*_*j*_	6
5	*ω*_*i*_ is extremely important than *ω*_*j*_	8
6	*ω*_*j*_ is slightly more important than *ω*_*i*_	1/2
7	*ω*_*j*_ is obviously more important than *ω*_*i*_	1/4
8	*ω*_*j*_ is more important than *ω*_*i*_	1/6
9	*ω*_*j*_ is extremely important than *ω*_*i*_	1/8

**Table 2:** Judgment parameter matrix.

	Production energy saving level	Ecological environmental protection level	Production emission reduction level
Production energy saving level	1	1/2	1/2
Ecological environmental protection level	2	1	1
Production emission reduction level	2	1	1

**Table 3:** Indicator weights.

Serial number	Indicator name	Weight
C1	Average energy consumption per workshop	0.022
C2	Average water consumption per workshop	0.081
C3	Average electricity consumption per workshop	0.045
C4	Elasticity of energy consumption in fish skin industry	0.012
C5	Local greening rate	0.105
C6	Workshop environmental protection	0.231
C7	Waste disposal rate	0.032
C8	Average wastewater discharge per workshop	0.135
C9	Average waste emissions per workshop	0.234
C10	Average exhaust emissions per workshop	0.072
C11	Industrial waste discharge compliance rate	0.019
C12	Industrial exhaust emission compliance rate	0.012

The article "Static and Dynamic Demonstration of the Ecological Level of Ethnic Cultural Industries Based on the Internet of Things and Environmental Responsibility" was retracted in 2023. Reasons: unreliable results or conclusions; concerns about the data; concerns about the peer review; concerns about the citations.

**Table 4:** Standards for classification of safety levels.

Security level	State	Score
E	Very dangerous	<0.3
D	Dangerous	[0.3,0.5)
C	Critical value	[0.5,0.7)
B	Safer	[0.7,0.9]
A	Very safe	>0.9

## Data Availability

The data that support the findings of this study are available from the corresponding author upon reasonable request.
